# Ecological Smart City Construction Based on Ecological Economy and Network Governance

This article has been retracted.

**DOI:** 10.1155/2022/5682965

**Published:** 2022-07-05

**Authors:** Yue Wu

**Affiliations:** University of New South Wales, High St, Kensington, Sydney, NSW 2052, Australia

## Abstract

China has paid huge resources and environmental costs in the rapid economic development, which severely restricts China's sustainable development. As a mesolevel between macro(state) and micro(enterprise), urban management has many features that are different from traditional management. This research mainly discusses the construction of ecological smart city based on ecological economy and network governance. This research analyzes the current situation and problems of urban construction from three aspects: urban ecological economy, urban ecological environment, and urban ecological society. The ecological indicators of smart cities are used to reflect the true situation of the target. In order to facilitate quantitative analysis with the greatest possibility and accuracy, a batch of representative, comprehensive, and quantifiable indicator data is the key. By drawing on the existing literature and implementing it under the circumstances, the selected methods are frequency analysis and theoretical analysis, which are divided into three parts: economy, environment, and society to construct an urban ecological evaluation index system. Under the new network governance environment, the openness of government affairs has become more transparent and time-effective. Moving the government's work to the network not only enhances the construction of a clean government, but also increases the level of public participation. The main ways of citizen participation created by network governance are carrying out online voting, making anonymous online speeches, and online inquiries about politics, etc. These ways have expanded the traditional government governance methods. Not only that, network governance can make the government's management process more transparent. In this situation, government activities are carried out under the supervision of citizens, which can alleviate the phenomenon of corruption. After the implementation of the ecological smart city plan, the green coverage rate of the built-up area of City A will increase by 1.8% compared with 2017, showing an upward trend. This research will provide effective guidance for the development of ecological smart cities.

## 1. Introduction

China's ecological city planning theory emphasizes ecological planning, ecological design, and ecological management. The theoretical research on ecological cities involves a lot of content. However, at present, the domestic ecology community has not been able to unite with the planning academia and other disciplines to carry out more influence.

It is necessary to conduct in-depth and systematic research on the application of comprehensive management of urban economic, social, and environmental systems. Starting from the study of the connotation and characteristics of ecological smart cities, this paper establishes an evaluation index system for ecological smart cities in China to more accurately evaluate the current development level of ecological smart cities in China and analyze the differences between ecological smart cities in different regions and the causes of differences [1, 2]. The reason is that it is easy to learn relevant advanced experience from it, then accurately locate various regions, find solutions to problems and improve strategies, and help builders grasp the direction of urban development, provide new impetus for sustainable urban development, and improve China's ecological wisdom construction level providing certain support. Based on the comparative study of urban governance theory and practice, this paper regards urban governance as a basic function of urban management, based on the self-organization mechanism of urban development and the system of urban board of directors.

Smart city is an advanced form of urban informatization after digital city and smart city, and it is a deep integration of informatization, industrialization, and urbanization. With the vigorous development and progress of the Internet of Things, smart cities have become an emerging paradigm, which consists of ubiquitous sensing, heterogeneous network infrastructure, and intelligent information processing and control systems. Zhang et al. believe that smart cities can monitor the physical world in real time and provide local residents and travelers with intelligent services in transportation, medical care, environment, entertainment, and energy. However, security and privacy issues follow, because smart city applications not only collect extensive privacy-sensitive information from people and their social circles, but also control city facilities and affect people's lives. He investigated the security and privacy in smart city applications. Specifically, he first introduced promising smart city applications and architectures. He then discusses several security and privacy challenges in these applications. He only investigated the security issues of smart cities and did not give an exact solution [3]. Menouar et al. believe that there is no smart city without a reliable and efficient transportation system. Although these two emerging technologies are critical to the realization of fully automated transportation systems, there is still a great need for the automation of other roads and transportation components. He described possible ITS applications where drones can be used and emphasized the potential and challenges of ITS that support drones in the next generation of smart cities. Although UAVs are envisioned for many ITS applications, the mobility, autonomous operation, and communication/processing capabilities are not very clear [4]. Sharma et al. (Pradip Kumar Sharma) believe that in recent decades the vehicle self-organizing network has become a core network technology that provides comfort and safety for drivers in the vehicle environment. However, emerging applications and services require major changes to the underlying network models and calculations that require new road network planning. He proposed a blockchain-based smart city car networking architecture (Block-VN). Block-VN is a reliable and secure architecture that runs in a distributed manner to build a new distributed transmission management system. He is considering building a new vehicle network system Block-VN on top of them. Although the blockchain in his research can be used to build an intelligent, safe, distributed, and autonomous transportation system, he did not give specific data for the research [5]. Brundu et al. introduced an IoT software infrastructure that supports new control policies for energy management and simulated urban areas. The proposed platform enables (near) real-time building energy profile interoperability and correlation with environmental data from sensors and building and grid models. In the smart city environment, the platform realizes the integration of heterogeneous data sources at the building and regional level, as well as the simulation of new energy policies at the regional level, with the aim of optimizing energy use and considering its impact on creating comfort. The platform has been deployed in a real area, and a novel heating network control strategy has been developed and tested. His research only explained the Internet of Things software but lacked the corresponding evaluation [6]. The city is the place where the reform achievements are the most prominent. Its most prominent feature is the various factors of production (the aggregation process of economic resources). For enterprises, in order to achieve the maximum utilization efficiency of production factors, it must operate with the purpose of maximizing economic benefits.

This research analyzes the current situation and problems of urban construction from three aspects: urban ecological economy, urban ecological environment, and urban ecological society. The ecological indicators of smart cities are used to reflect the true situation of the target. In order to facilitate quantitative analysis with the greatest possibility and accuracy, a batch of representative, comprehensive, and quantifiable indicator data is the key. By drawing on the existing literature and implementing it under the circumstances, the selected methods are frequency analysis and theoretical analysis, which are divided into three parts: economy, environment, and society to construct an urban ecological evaluation index system. In the process of urban development, it is necessary to comprehensively manage economic, social, and environmental factors and coordinate the relationship between all aspects.

## 2. Research Method

### 2.1. Network Governance

The continuous development and progress of network information technology have posed new challenges to traditional public management. Nongovernmental departments and government departments should adhere to the governance concept of interdependence and mutual cooperation (network relationship), and take collective actions on issues of common concern. In the process of modern social governance, traditional social governance concepts can no longer meet the needs of modern residents, and the concept of network governance was born. Network governance theory embodies the governance of people on the network. In order to achieve governance goals, network governance theory believes that many temporary relationships should be built to realize public decisions within a specific network and all the governors and participants must be integrated into a specific network. In the process of network governance, the administrator builds a specific network and provides management and services in the specific network. However, due to the diversification of network participants, the government may only be the main body of a particular network unit and may not be the main body or the only main body in another network. This network only provides the means for all parties to communicate directly. Platform and the degree of participation of netizens and the degree of trust and compliance with government administrative actions are the key to the smooth operation of governance [7].

“Smart city” integrates the elements of the original city concept, such as urban management, business activities, culture and education, transportation and logistics, health care, and energy resources, through the extensive use of Internet of Things, cloud computing, big data, and other network technologies, in accordance with more modern, networked urban development concept, deep integration of existing important projects, so that governors have a quick response to the city's convenience services, public governance, public security and stability, transportation and logistics, people's livelihood, and commerce and continuously improve urban construction. Planning, service management, and networking of production and life make urban production and life management faster and greener [8–10]. It is an upgrade to the original urban system. In the planning and construction, hardware and software must be available, and the software environment and hardware equipment must be developed together to make the city's various systems more harmonious and intelligent, so that residents living in smart cities will have more gains. Through a sense of belonging, life is more comfortable and pleasant [11].

The penalty function, also known as the penalty function, is a type of constraint function. For constrained nonlinear programming, its constraint function is called a penalty function, and its parameter is called a penalty factor (or penalty parameter). Assuming that x_j_ is the *j*-th index data and x_max_ is the maximum value of the *j-*th index, the normalized value of the positive index is [12].

(1) $$\begin{array}{c} {\text{x}}_{ij}=\frac{\left(x_{j}-x_{\min}\right)}{\left(x_{\max}-x_{\min}\right)}. \end{array}$$

The standardized value of the negative indicator is [13]

(2) $$\begin{array}{c} {\text{x}}_{\text{ji}}=\frac{\left(x_{\min}-x_{j}\right)}{\left(x_{\max}-x_{\min}\right)}. \end{array}$$

Network governance itself has strong tool attributes, and it can realize a way different from traditional governance methods with the help of electronic means. Under the new network governance environment, the openness of government affairs has become more transparent and time-effective. Moving the government's work to the network not only enhances the construction of a clean government, but also increases the level of public participation. The main ways of citizen participation created by network governance are carrying out online voting, making anonymous online speeches, and online inquiries about politics, etc. These ways have expanded the traditional government governance methods. Not only that, network governance can make the government's management process more transparent. In this situation, the government's activities are carried out under the supervision of citizens, which can alleviate the phenomenon of corruption and truly achieve power in the sun.

Let the sample set *A*={(x,*y*), *x* ∈ *R*} introduce the nonnegative slack variable *ξ* and the penalty factor C [14]:

(3) $$\begin{array}{c} Y-\omega^{T}\phi \left({\text{x}}_{i}\right)-b\leq \varepsilon +\xi . \end{array}$$

Therefore, integration should be the biggest feature of urban construction smart complexes. It should cover social services such as smart city services, smart medical care, smart business, smart home, and smart security, to maximize service efficiency. In order to alleviate the pressure of government investment and improve the efficiency of urban smart city construction, the government should change the service concept and introduce more enterprises, social organizations, and residents [15, 16]. On the one hand, various channels, such as centralized training for street and smart city staff, actively promote the application of smart platforms, so that everyone can quickly learn and adapt to new management methods and communication models. On the other hand, enterprises activate the smart city construction market with social organizations, streamline administration, and delegate power, integrate resources, and let more professionals and organizations do more professional things and at the same time actively promote the sustainable development of smart cities by optimizing the functions of smart platforms. Let smart cities meet the needs of residents' daily lives and allow smart city residents to actually experience the convenience brought by wisdom [17–19].  Figure 1 shows the network governance of an ecological smart city.

### 2.2. Principles for Selection of Ecological Smart City Indicators

The time and space perspectives of smart cities are very large, ranging from economic efficiency and efficiency to life-level transportation, tourism, elderly care, and medical care, as well as high-level planning and smart industries. The conditions of each city are very different, and the development model and construction focus are also different. It is necessary to adjust measures to local conditions and formulate suitable construction paths. When constructing a smart city ecological evaluation index system, it is impossible to establish a set of indicators for each city. If this is the case, it lacks the ability of comparison horizontally. Through the analysis of the existing literature, we can learn from its merits, in order to achieve the highest degree of recognition of the indicators. There are several rules for constructing a smart city ecological evaluation index system [20].

#### 2.2.1. Scientific Evaluation

In order to have a scientific and objective evaluation of urban ecological construction, the index system must follow scientific principles, faithfully reflect the connotation and basic principles of urban ecological construction, and consider both economic growth and environmental protection, and the selection of data must be based on authentic sources and use standards.

#### 2.2.2. Operability

If the operability of the index system is not strong, it will cause a lot of inconvenience in subsequent use. Maneuverability requires that the index system be practically useable. First of all, from an ecological perspective, the index system is quite extensive, and the economic feasibility and cost-effectiveness of data collection must be taken into consideration. Second, the index system can be quantified. Only after the index is quantified, can the next step of comparison be entered. This is the purpose of the final analysis. Finally, the indicators must be consistent with the measurement target and can truly reflect the status of the measurement target.

#### 2.2.3. Comparability

The principle of comparability requires that the index system can be used between different cities in order to evaluate and analyze the results. In the process of data collection, some index data is quite difficult, so it is necessary to find its substitute index or delete the index.

#### 2.2.4. Combination of Ecology and Economy

The design of the indicator system for the ecological construction of smart cities should fully reflect the characteristics of ecology and reflect the ecological characteristics of the city. In addition, the development of cities cannot be separated from rapid economic growth and human progress. Therefore, the indicator system has to reflect the economic side. In other words, the evaluation index must meet both the ecological requirements and the service requirements for economic development.  Figure 2 shows the realization process of an ecological smart city.

### 2.3. Building an Indicator System

The ecological indicators of smart cities are used to reflect the true situation of the target. In order to facilitate quantitative analysis with the greatest possibility and accuracy, a batch of representative, comprehensive, and quantifiable indicator data is the key. By drawing on the existing literature and implementing it according to the situation, the selected methods are frequency analysis and theoretical analysis, which are divided into three parts: economy, environment, and society to construct an urban ecological evaluation index system [21].

#### 2.3.1. Frequency Analysis Method

Carefully study the information on the urban ecological evaluation index system in the existing master and doctoral dissertations and journal literature and carefully count the indicators used and displayed in tables. When an indicator is used more easily, it will be easily accepted, and its frequency of occurrence accordingly will be bigger. Therefore, this article chooses the top-ranked indicators as much as possible, so that the establishment of the indicators has a basis and reference.

#### 2.3.2. Theoretical Analysis Method

Perform a secondary analysis of the indicators initially selected by the frequency statistics method, combined with the characteristics of ecological economics and analyze the three major levels of economy, environment, and society. According to the actual situation, delete inappropriate indicators, add, or modify some indicators, so that it can reflect the reality and the operation to be simple. The first step is the frequency analysis method. There are 33 documents involved in the statistics, including 23 dissertations and 12 journal papers, and carefully record various indicators related to ecological evaluation to ensure accuracy and no omissions. The second step is to carry out the theory. Analyze and fully consider the ecological economic integration of ecological economics, under the premise of satisfying the principle of index construction, the availability, and applicability of comprehensive index data collection; some statistical results are shown in Table 1.

Fine particulate matter refers to particulate matter with aerodynamic equivalent diameter less than or equal to 2.5 microns in ambient air. Both PM10 and PM2.5 are measures of inhalable particulate matter. However, in recent years, due to the seriousness of air pollution, people have increasingly incorporated pollution issues into private decision-making. However, China's monitoring standards and monitoring content in this regard are not yet perfect. Monitoring methods and punishment measures are not perfect; operability and implementability are poor, so this article will not consider this indicator. The harmless treatment rate of industrial solid waste and the treatment rate of industrial solid waste are unified into the comprehensive utilization rate of industrial solid waste. Taking into account the convenience of statistical data, the general predetermined income of local finance is included in the per capita fiscal revenue, and the afforestation area and the coverage rate of garden green land in the year are included in the per capita public green area. The number of hospital beds per 10,000 people and the number of licensed doctors per 1,000 people are used to measure the basic level of medical care in a city. In view of the repeatability and the difficulty of obtaining data, the number of doctors per 10,000 people is a uniform indicator. The proportion of employment in the tertiary industry is included in the proportion of tertiary industry in GDP, and the per capita net income of residents is included in the annual per capita disposable income of residents [22]. GDP (gross domestic product) is the final result of the production activities of all resident units in a country (or region) within a certain period of time.

Standardize the initial index data and set the standardized value of each index data to *Y* [23]:

(4) $$\begin{array}{c} Y=\frac{x_{ij}-\min\left(x_{i}\right)}{\text{max}\left(x_{i}\right)-\text{min}\left(x_{j}\right)}. \end{array}$$

Calculate the information entropy value of each indicator; the information entropy value of the j-th group of indicator data is [24]

(5) $$\begin{array}{c} S=-\text{ln}{\left(n\right)}^{-2}\sum_{1}p. \end{array}$$

Among them,

(6) $$\begin{array}{c} \text{p}=\frac{y}{\sum_{i=1}^{n}Y}. \end{array}$$

For the index weight vector [25],

(7) $$\begin{array}{c} \text{p}=\frac{y}{\sum_{i=1}^{n}Y}. \end{array}$$

Among them,

(8) $$\begin{array}{c} {\text{w}}_{j}=\frac{\left(1-S\right)}{\sum_{j=1}^{m}S,0\leq W\leq 1}. \end{array}$$

### 2.4. Determination of the Evaluation Index System

The existing ecological evaluation indicators basically focus on two levels. One is to consider the ecological niche and analyze the ecological situation and development of the city from the three perspectives of biological niche, organizational niche, and urban niche. The other is to divide the city into three subsystems: nature, society, and economy. The difference between these two classification methods is mainly that the second-level and third-level indicators are different, but the underlying indicators are similar. Considering that the three major aspects of urban construction are economy, environment, and society, this classification can analyze the current situation and problems of urban construction at a glance. So, this article is analyzed from three aspects: urban ecological economy, urban ecological environment, and urban ecological society. Among them, the economy is the foundation of urban development, and a good economic level and optimized economic structure are the keys to the balanced development of various subsystems of the city; the ecological environment is the basis for economic development, and the function of the ecological environment system supports the development of the economic system and humanity. The survival of the city, the greening of the city, the quality of the environment, and the degree of environmental governance are closely related to our lives; the ecological society mainly refers to the perfection of the infrastructure used by people and development opportunities [26]. Part of the urban ecological evaluation index system constructed in this paper is shown in Table 2.

The test statistics is

(9) $$\begin{array}{c} \gamma^{2}=\text{m}\left(n-1\right)F. \end{array}$$

The construction of a smart city must rely on the development foundation and humanistic environment of the city. It is necessary not only to build a high-rise building to do a good job in the overall planning, but also to proceed from the actual situation of the city, in most cases subject to *γ*^2^(n − 1) [27]:

(10) $$\begin{array}{c} F=\frac{\sum_{\text{i}=1}^{n}R^{2}-3mn\left(n+1\right)}{mn\left(n^{2}-1\right)}. \end{array}$$

R is the sum of the ratings of each evaluation object [28]. Assumptions are the following:

(11) $$\begin{array}{c} \gamma^{2}\geq \gamma^{2}\left(\text{n}-1\right). \end{array}$$

It is considered that the evaluation grades of *m* kinds of evaluation methods are consistent; otherwise, they are not consistent. The final evaluation value is obtained by weighted summation of *p* principal components, and the weight is the variance contribution rate of each principal component [29]:

(12) $$\begin{array}{c} \alpha =\frac{\lambda }{\sum_{\text{i}=1}^{p}\lambda_{j},j=1,2,\ldots ,p}. \end{array}$$

Final evaluation [30]:

(13) $$\begin{array}{c} F=\sum_{\text{i}=1}^{k}\alpha F_{n},n=1,2,\ldots ,p. \end{array}$$

## 3. Results

Using the multistatistical source data of the four cities (City A, City B, City C, and City D) in 2020 as the original data, the factors that have a cumulative variance contribution rate of over 85% are selected to construct a factor score coefficient matrix. The variance contribution rate corresponding to the factor is a weight, which is substituted into the comprehensive evaluation formula F to obtain the comprehensive score and ranking of the sample city, which provides data support for the subsequent analysis of the reasons. The original data of the four cities are shown in Table 3.

It can be seen from Figure 3 that the ranking results of economic indicators are City B, City C, City A, and City D. City B has the highest comprehensive score for smart economy indicators, indicating that City B's smart economy is better developed than the other three cities. City A is in the third place. It is relatively low in terms of per capita gross regional output value and urban per capita disposable income. There is still a lot of room for economic growth, and it must play its own expertise in attracting capital investment. Develop high-tech industries, promote the transformation and upgrading of traditional heavy industries, and promote stable economic growth. The comparison of scientific and technological indicators is shown in Figure 3.

It can be seen from Figure 4 that City C has the highest comprehensive score of smart ecology and smart people's livelihood indicators. The order of the four cities is C city, A city, *D* city, and B city. The comprehensive score of the economic indicator system of City A is 0.08, ranking second. The green coverage rate in the built-up area of City A is the lowest among the four cities, only 33.7%, which is 10.2% different from City C. The harmless treatment rate of domestic waste is also ranked the lowest among the four cities. Environmental protection and capital investment should be increased, and industrial waste should be discharged after qualified treatment, and vigorously develop an environmentally and friendly economy. A good urban environment can promote the construction of smart cities and improve the public's sense of happiness and experience. Among the two indicators of the number of beds in medical institutions per 1,000 people and public toilets (class three), City A ranks the first, and the number of buses and trams per 10,000 people is second only to City C, which ranks the first. The indicators of smart ecology and smart people's livelihood are shown in Figure 4.

Figure 5 shows that the comprehensive evaluation rankings of the four cities are City C, City B, City A, and City D. The F1 index score is higher in City C, the F2 index score is highest in City B, the F3 index score is highest in City A, and City C has the highest comprehensive score. Compared with other cities with similar economic structures, City A still has a lot of room for development. The gap in economic aggregates is obvious, and there are many constraints in infrastructure construction and urban environmental protection. We must pay attention to the cultivation of scientific and technological talents and adopt a development model that combines production, learning, and research to lay a solid material foundation for the construction of smart cities. The comprehensive evaluation of smart cities is shown in Figure 5.

For the four indicators of per capita regional product, urban per capita disposable income, rural per capita disposable income, and total post and telecommunications business, there is an overall upward trend from 2017 to 2020, and the total post and telecommunications business will break a new high of 242.9 in 2020, 100 million yuan, which is 1.735 times that of 2017. For the indicator of fixed asset investment, in the middle of 2017–2020, this indicator has shown an upward trend as a whole. In 2020, compared with 2017, there was the overall increase of 121.95 billion yuan.  Figure 6 shows the division of assets in different quarters.

It can be seen from Figure 7 that the green coverage rate in the built-up area of City A has increased by 1.8% compared with 2017, showing an upward trend. For the three indicators of comprehensive utilization of industrial solid waste, per capita park, green area, and urban sewage treatment rate, there will be an upward trend from 2020 to 2020. The three indicators are all positive indicators. The larger the value, the greater the degree of environmental protection, which is favorable. For the indicator of the number of days with good air quality, the overall trend from 2020 to 2020 shows a first decline and then an upward trend. There is a certain decline in 2018 and 2020. The number of days with good air quality in 2019 reached the highest value of 282 days. The year 2020 is 227 days, with a large gap and obvious fluctuations. For the indicator of per capita park and green area, there will be no significant changes from 2020 to 2020, and both are 9 to 10 persons per square meter. In 2020, the per capita park and green area will reach the highest value of 10.9 persons per square meter. In general, in terms of smart ecology, in the four years from 2020 to 2020, the smart ecology level of City A is developing in a positive direction. The smart ecological evaluation is shown in Figure 7.

## 4. Discussion

The government is a planner and participant in the construction of smart cities. It should reasonably set the development goals of various fields and departments, formulate short-term, medium-term, and long-term development plans, formulate and issue various supporting policies to promote urban development, and provide financial, material, and intellectual resources. Pay attention to cross-city, cross-department, communication, and cooperation between government, enterprise, and people to systematize the management system and break the traditional block-based political system. Accelerate the construction of urban big data and cloud platforms, create a city-wide information sharing platform, promote city-wide information data sharing and integration, improve information network security awareness and resistance, and create a good environment for coconstruction and sharing [31, 32].

Smart city is a brand-new grassroots governance method, which is closely related to local humanities, geography, environment, culture, government, residents, and other elements. The construction of smart cities is not just a simple transformation and upgrading of traditional smart cities. It cannot be achieved by introducing smart city platforms. This is a long-term investment process. Network technology, hardware facilities, government agencies, policy support, standards, and regulations only by organically combining with the evaluation system and other hardware foundations and the humanistic environment, historical foundation and other soft conditions, can we build a smart city system with city characteristics. It is necessary to integrate the actual conditions of city, including government administration, administrative regulations, convenient facilities, humanistic level, residents' autonomy, and self-quality and increase investment in all aspects of resources such as infrastructure, technological innovation, residents' quality, and government concepts, in order to realize the construction of smart cities [33]. The country is currently comprehensively promoting the rural revitalization strategy, which is a complex overall strategy. This paper takes smart city as an example; through field surveys and visits and data collection analysis, the construction and governance of smart cities are researched and summarized. In addition, it is necessary to improve the community governance system, give full play to the government's dominant position in social management at the source, plan the overall situation, continuously train information and community management professional management personnel, improve the cultural quality of smart city residents, and promptly resolve the development of smart cities various risks encountered in development [34, 35]. Networked governance is not only a brand-new analytical tool, but also a governance model that challenges the traditional government system, representing a profound understanding of governance subjects, governance tools, governance structures, and governance mechanisms' change.

Based on the research of relevant theories at home and abroad, the summary of previous research results, and the analysis of their connotations, this research summarizes the evaluation systems of ecological cities, smart cities, and ecological smart cities and constructs an ecological smart city evaluation that meets the current situation in China. The system can provide support for the government to do a good job in item-level design. The design of an ecological smart city evaluation model has built a bridge for the development of China's ecological smart city from theory to practical operation [36]. The research in this paper on the theoretical basis of the development process, connotation, and subject of the ecological smart city can enable the subjects to have a deeper understanding of the essence and development positioning of the ecological smart city [37]. The construction of the evaluation model has built a bridge for the development of China's ecological smart city from theory to practical operation. It can enable cities and regions to fully understand their own advantages and disadvantages in various aspects and can adapt to local conditions and combine their own actual conditions to give full play to their own advantages. The formulation of action plans and development directions promote the transformation and upgrading of urban construction models to the direction of “ecology + wisdom” and has important practical significance for the reasonable and efficient allocation of urban resources in the construction of ecological smart cities in China and the improvement of urban livability [38, 39].

## 5. Conclusion

This research analyzes the status quo and problems of urban construction from three aspects: urban ecological economy, urban ecological environment, and urban ecological society. Under the new network governance environment, the openness of government affairs has become more transparent and time-effective. Moving the government's work to the network not only enhances the construction of a clean government, but also increases the level of public participation. This research will provide effective guidance for the development of ecological smart cities. Present the relevant models of networked governance, clarify the essential connotation of networked governance, and list the theoretical research of networked governance at different levels. After comparing and improving the indicators, we can consider diverse evaluation methods and decision-making methods and use more objective data analysis methods to reflect the construction and development of smart ecological cities, so as to better avoid system errors caused by experts' subjective evaluations. Make more detailed and accurate evaluation for the evaluation object and improve the evaluation accuracy. Networked governance is a new form of government governance, which promotes the degree of socialization, flattening, and specialization of government governance. In the future work, the evaluation index system of the smart city monitoring and control system can get the attention of relevant departments or be promoted and applied. In practice, it is combined with the development of sponge facilities in various regions to develop a monitoring and control system for smart ecological cities in various regions according to local conditions. The evaluation system and the establishment of a complete feedback correction mechanism in the application process can truly be used to manage sponge cities, improve management efficiency, and realize the significance and value of this research.

## Figures and Tables

**Figure 1:** Network governance of ecological smart cities.

**Figure 2:** The realization process of ecological smart city.

**Figure 3:** Comparison of technological indicators.

**Figure 4:** Smart ecology and smart livelihood indicators.

**Figure 5:** Comprehensive evaluation of smart cities.

**Figure 6:** Asset division in different quarters.

**Figure 7:** Smart ecological evaluation.

**Table 1:** Some statistical results.

Project	Unit	Frequency	Relative frequency (%)
PM2.5 indicator	—	12	34.28
Water consumption per unit GDP	m^2^/ten thousand yuan	12	34.28
The number of days with air quality above grade II accounted for the proportion of the whole year	%	12	34.28
Industrial water reuse rate	%	12	34.28
Per capita fiscal revenue	Ten thousand yuan	10	28.57
The proportion of total fixed asset investment in GDP	%	8	22.8
Public transportation vehicles per 10,000 people	Vehicles	7	20
Drinking water source quality compliance rate	%	3	8.57
Urbanization rate	%	3	8.57

**Table 2:** Part of the urban ecological evaluation index system constructed in this paper.

First level indicator	Secondary indicators	Three-level indicators
Urban ecological construction	Urban ecoeconomic system	GDP per capita
		GDP growth rate
		Local fiscal revenue
	Urban ecological environment system	Green coverage rate in built-up area
		Urban public green area per capita
		Harmless treatment rate of domestic garbage
	Urban ecological social system	Natural population growth rate
		Urban registered unemployment rate
		Passenger volume

**Table 3:** Raw data of four cities.

Variable	City A	City B	City C	City D
Green coverage rate in built-up area (%)	42.1	43.9	33.7	41.5
Number of days with good air quality (days)	256	300	270	276
Park and green area per capita (person/square meter)	127	11 3	10.9	1075
Comprehensive utilization rate of industrial solid waste (%)	79	77.84	95.16	70.7
Urban sewage treatment rate (%)	94.2	94	96	95
Harmless treatment rate of domestic garbage (%)	87	100	100	89
Number of beds in medical institutions per thousand population (pieces)	8 58	8 37	6.57	6.66
Public toilets (above category three)	951	550	345	767
Public library collections (thousand volumes)	5774	5661	10339	5650

## Data Availability

The data that support the findings of this study are available from the corresponding author upon reasonable request.
